This article has been retracted.

# Effect of Minimally Invasive Puncture Drainage and Conservative Treatment on Prognosis of Patients with Cerebral Hemorrhage

**DOI:** 10.1155/2021/2401256

**Published:** 2021-12-23

**Authors:** Yanxun Jia, Yongbin Wang, Kaijiao Yang, Rui Yang, Zhenzhen Wang

**Affiliations:** ^1^Department of Neurosurgery, Eighth People's Hospital of Hengshui City, Hengshui 253800, China; ^2^Department of Neurology, Eighth People's Hospital of Hengshui City, Hengshui 253800, China

## Abstract

The objective of this study was to explore the effect of minimally invasive puncture drainage under unsupervised learning algorithm and conservative treatment on the prognosis of patients with cerebral hemorrhage. Fifty patients with cerebral hemorrhage were selected as the research objects. The CT images of patients were segmented by unsupervised learning algorithm, and the application value of unsupervised learning algorithm on CT images of patients with cerebral hemorrhage was evaluated. According to the treatment wishes of the patients themselves and their authorizers, they were divided into 30 patients with cerebral hemorrhage in the minimally invasive group and 20 patients with cerebral hemorrhage in the conservative group. The incidence rate of complications of cerebral hemorrhage, the length of hospitalization of the two groups, hematoma volume at admission, 3 days and 7 days after operation, and the hematoma dissipation rate on the 3rd and 7th day after operation were used as the evaluation index of therapeutic effect. MRS and ADL scores were used as prognostic indicators. The results show that *K*-means clustering algorithm has high quality and short time for CT image segmentation. The overall incidence rate of complications in minimally invasive group was 10%, lower than that in conservative group (25%) (*P* < 0.05), and the length of hospitalization in minimally invasive group was longer than that in conservative group (*P* < 0.05). The hematoma volume of minimally invasive group was 16.5 ± 2.4 mL on the 3rd day after operation, and that of conservative group was 27.4 ± 1.8 mL. There was significant difference between the two groups (*P* < 0.05). In addition, CT showed that the hematoma reduction degree of minimally invasive group was higher than that of conservative group, and the hematoma dissipation rate was higher than that of conservative group on the 3rd and 7th day (*P* < 0.05). The good MRS score in minimally invasive group was 3.15 times that in conservative group, and the good ADL score was 1.6 times that in conservative group, and there was significant difference in the total score between the two groups (*P* < 0.05). Minimally invasive puncture drainage is better than conservative treatment in the clearance of hematoma, which is conducive to the recovery of neurological function and daily life of patients with cerebral hemorrhage and is of great help to the prognosis of patients.

## 1. Introduction

The definition of cerebral hemorrhage refers to the cerebral parenchymal hemorrhage caused by nontrauma. It is a common brain disease in neurology and belongs to stroke subtype [1]. Cerebral hemorrhage is usually due to the patient's own basic hypertension disease, combined with arteriosclerosis. Two disease factors promote cerebral hemorrhage [2, 3]. The pathology of cerebral hemorrhage mainly comes from cerebral arteries such as the anterior cranial artery, the middle cranial artery, the posterior cranial artery, and the perforator artery in the brain stem. Under the pressure of the patient's own hypertension, some degenerative pathological changes have taken place in the arterial wall of the cranial artery, including the arterial middle membrane and arterial smooth muscle, which is finally manifested as the patient's sudden craniocerebral hemorrhage [4, 5]. The method of dealing with primary injury can only control and not expand hematoma, but it cannot improve the nerve damage. The injury after cerebral hemorrhage is the inflammatory factors and cytotoxicity produced by the hematoma itself and/or its released substances. These two substances will cause secondary edema in the surrounding tissues of the hematoma, also known as edema around the hematoma. Edema around the hematoma is an important link of cerebral hemorrhage, and so many scholars regard it as the key to the treatment of cerebral hemorrhage [6, 7].

Although the traditional craniotomy evacuation of hematoma can remove hematoma, but because the trauma is relatively large, more postoperative complications occur to patients with subsequent secondary injury [8, 9]. The use of minimally invasive puncture drainage for the treatment of cerebral hemorrhage is gradually attracting people's attention. Minimally invasive puncture drainage is to successfully locate the hematoma in the brain by means of imaging and then effectively remove the hematoma by using liquefied agent and suction equipment [10]. Clinical studies have found that minimally invasive puncture drainage in the treatment of cerebral hemorrhage can accelerate the removal of intracranial hematoma time, reduce intracranial pressure, control the development of cerebral hemorrhage as soon as possible, and prevent the prognosis of complications, so as to effectively reduce the mortality of cerebral hemorrhage, prolong the life of patients with cerebral hemorrhage, and improve the quality of life [11]. Although minimally invasive puncture drainage is an effective treatment for most patients with cerebral hemorrhage, the prognosis of patients is not clear.

With the rapid development of computer technology and medical information, unsupervised learning algorithm plays a great role in clinical application in helping imaging doctors to mine more in-depth and detailed imaging information of patients. It can deeply analyze image data and has been applied to the prediction of disease incidence and prognosis. Unsupervised learning algorithm is generally divided into clustering algorithm and dimension reduction algorithm, including clustering algorithm, hierarchical clustering algorithm, density-based clustering kernel function algorithm, density-based clustering deep neural network algorithm, principal component analysis, independent component analysis, distributed domain embedded algorithm, and other algorithms. However, the *K*-means clustering algorithm is one of the most classical clustering algorithms. The *K*-means clustering algorithm can segment the lesion of the imaging image. Through the reasonable mining of the image data and the correct analysis of the lesion area, the three-dimensional framework of the medical image of the lesion or the feature area can be reconstructed to assist clinicians in formulating more accurate treatment plans [12].

Based on this, the patients with cerebral hemorrhage were grouped by minimally invasive puncture drainage and conventional conservative treatment through retrospective analysis. The application value of *K*-means clustering algorithm in CT images of patients with cerebral hemorrhage was evaluated. The effects of the two groups on the improvement of cerebral hemorrhage and the prognosis of patients on the 3rd and 7th day after admission were compared, so as to provide reference for doctors to choose reasonable treatment methods for patients in clinical treatment.

## 2. Methods

### 2.1. Research Objects

50 patients with cerebral hemorrhage admitted to the Department of Neurosurgery of XX Hospital from January 2020 to July 2021 were selected as the research subjects. According to the patient himself and the patient's authorization, 50 patients were randomly divided into minimally invasive group and conservative group. In the minimally invasive group, there were 30 cases, 18 males and 12 females, aged between 26 and 59 years, with an average age of 42.5 years. In the conservative group, there were 20 cases, 11 male patients, 9 female patients, aged between 29 to 60 years, with an average of 44.5 years old. Consciousness level standard was divided into fully awake, drowsy or hazy, and drowsy. There was no significant difference between the two groups in general data, including age, gender, onset time of cerebral hemorrhage, history of hypertension, bleeding volume, and consciousness status classification (*P* > 0.05), which can be used for subsequent comparison.

  Inclusion criteria: (1) patients in the two groups were aged from 26 to 59 years; (2) the diagnosis was confirmed as cerebral hemorrhage according to the 2019 Edition of *Chinese Guidelines for the Diagnosis and Treatment of Cerebral Hemorrhage*, and the diagnosis was confirmed as cerebral hemorrhage by imaging examination; (3) all patients had a history of hypertension; (4) all patients received treatment for the first time at admission, and the onset time was less than 24 hours; (5) the degree of disease can accept conventional conservative treatment; (6) the maximum amount of brain bleeding was 30 mL; (7) no liver, kidney, and other important organ dysfunction diseases were present.
  Exclusion criteria: (1) the patients were aged under 26 or over 60 years; (2) the presence of serious coagulation dysfunction or long-term use of anticoagulant drugs; (3) there was another secondary cerebral hemorrhage, such as cerebral hemorrhage caused by trauma, aneurysm, brain tumor, and stroke; (4) the patient's pathological data and imaging data within 24 hours of hemorrhage were incomplete.

All patients in this study or their authorized family members have signed informed consent, and the study program has been approved by the Medical Ethics Committee of XXX Hospital.

### 2.2. Treatment Methods

Treatment of minimally invasive group: the operation was performed within 12 hours of onset. All the operations were carried out in the intensive care unit by suctioning hematoma and drainage of liquefaction agents. The patients were anesthetized by 2% lidocaine. Before the operation, the head CT scanning was used to locate the hematoma in the brain to determine the center of the hematoma, the puncture position of the head, and the optimal puncture path. The puncture point was 10 cm from the nasal root and 4 cm from the middle line of the same side of the hematoma. The YL-1 intracranial puncture needle was used to puncture the hematoma and put into the 12th drainage tube. If a dark red liquid outflow was found, it was proved that the puncture needle had entered the hematoma, and 0.6 cm inward along the direction, ensuring that it did not exceed the specified puncture depth. When the drainage process was observed to be smooth, the tube core was removed, and then a disposable sterile syringe was used to slowly suction the hematoma, and suction should be less than 55%. After the operation, 5 mL of normal saline was used to clean the hematoma cavity every day, and 10 × 10^3^ IU/mL urokinase was injected to promote the dissolution of the remaining blood mass. The drainage tube was clamped for 2 hours and then the drainage was opened. The drainage was fixed 1–3 times a day. The volume of hematoma is generally less than 5 mL or disappears in about 3-5 days. When the hematoma disappeared, the drainage tube was pulled out. CT examination was performed on the 3rd and 7th days after operation.

Conventional conservative treatment: in the group of patients only given the prescribed medical conservative treatment, the patient's vital signs were monitored in real time, the patient's blood pressure was stable, the amount of water was stable, the electrolyte balance in the body was balanced, and the dehydration was carried out conservatively to reduce intracranial pressure. The proton pump inhibitor was used to protect the gastrointestinal mucosa, and the appropriate antibiotics was used to prevent infection.

### 2.3. *K*-Means Clustering Analysis Based on Unsupervised Learning Algorithm

Among the classical clustering algorithms in unsupervised learning algorithms, *K*-means clustering analysis is one of the most commonly used clustering algorithms in current literature. *K*-means clustering algorithm is a continuous iterative algorithm to adjust the clustering center, generally Euclidean distance as a similarity index. It takes the sum of the distance from the data point to the cluster center as an improved objective function and then uses the extreme value calculation method of this function to obtain the iterative operation rules. In this study, two-dimensional maximum entropy algorithm and *K*-means clustering algorithm were used to compare the CT image quality of patients with cerebral hemorrhage and the average time consumption of image segmentation. The basic principle of *K*-means clustering algorithm is as follows:

(1) $$\begin{array}{c} W=\overset{n}{\underset{i=1}{\sum }}\underset{j\in A_{i}}{\sum }{\left|j-\mu_{i}\right|}_{2}^{2}, \end{array}$$

where *μ*_*i*_ represents the mean vector of cluster *i* and its function equation is as follows:

(2) $$\begin{array}{c} \mu_{i}=\frac{1}{\left|X_{i}\right|}\sum_{j\in A_{i}}j. \end{array}$$

### 2.4. Observation Indicators of Therapeutic Efficacy

We used the following four indicators as efficacy indicators: (1) the incidence of complications in two groups of patients, as this study specifically refers to intracranial infection, pulmonary infection, and bleeding; (2) length of hospital stay of the two groups; (3) the hematoma dissipation rates of the two groups on the 3rd and 7th postoperative days calculated as shown in (3); (4) craniocerebral hematoma volume of patients in the two groups before admission, on the 3rd day after operation, and on the 7th day after operation: in this study, the multifield equation was used. For example, the amount of bleeding calculated by (4) can be used as one of the relatively simple independent factors for the prognosis evaluation of cerebral hemorrhage. Therefore, the volume measurement of craniocerebral hematoma plays an important role in the clinical formulation of treatment plans.

(3) $$\begin{array}{c} S=\frac{A-B}{A}\times 100\%, \end{array}$$

(4) $$\begin{array}{c} V=R\times W\times \delta , \end{array}$$

where *A* represents the amount of hematoma before treatment, *B* represents hematoma volume after treatment, *R* represents the radius of hematoma, *W* represents the width of hematoma, and *δ* represents the thickness of hematoma.

### 2.5. Prognostic Evaluation Indicators

All patients were followed up by telephone and regular outpatient. The prognosis was evaluated by modified Rankin Scale (MRS) and activities of daily living (ADL). The MRS score level and ADL score level are scored according to Table 1.

### 2.6. Statistical Analysis

All data of this study are analyzed by SPSS20.0 statistical software. The measurement data are expressed as mean ± standard deviation ($\bar{X}$ ± *s*), and the independent *t* test is used for the comparison between the two groups. The counting data are expressed in percentage (%). When *P* < 0.05, it is considered that the difference is significant and statistically significant.

## 3. Results

### 3.1. Basic Data of Two Groups of Patients

In this study, 50 patients with cerebral hemorrhage were selected as the research object. There were 30 cases in the minimally invasive puncture drainage group and 20 cases in the conventional conservative treatment group. According to the factors that may affect the prognosis of cerebral hemorrhage, the factors of the two groups were compared. The results showed that there was no significant difference between the two groups (*P* > 0.05), as shown in Table 2.

### 3.2. Segmentation Index Results of Unsupervised Learning Algorithm on CT Images

The *K*-means clustering algorithm is used to segment the lesion region of CT images of patients with cerebral hemorrhage. The segmentation result is shown in Figure 1. It is clearly evident from Figure 1 that the segmentation quality of *K*-means clustering is better than that of two-dimensional maximum entropy algorithm, the segmented lesions are clear, the range positioning of lesion location is more accurate, and the resolution is higher, and the average time consumption of *K*-means clustering algorithm is 0.96 s, which is shorter than that of two-dimensional maximum entropy algorithm by 1.05 s. It is suggested that *K*-means clustering algorithm has higher application value in the extraction and segmentation of lesion sites on CT images of patients with cerebral hemorrhage.

### 3.3. Comparison of Complications and Length of Stay between the Two Groups

The length of stay in the minimally invasive group was 10 ± 1.2 days and that in the conservative group was 18 ± 2.4 days as shown in Table 3. The length of stay in the minimally invasive group was significantly longer than that in the conservative group (*P* < 0.05). The incidence of complications in the minimally invasive group was 10%, lower than 25% in the conservative group (*P* < 0.05), but the independent incidence rate of complications was not significant.

### 3.4. Hematoma Dissipation Rate of the Two Groups after Operation

The hematoma dissipation rates of the two groups on the 3rd and 7th day after operation were compared. According to the figure, the hematoma dissipation rate in the minimally invasive group was 48.9% on the 3rd day after operation, the hematoma clearance rate on the 7th day was 83.6%, the hematoma dissipation rate in the conservative treatment group was 16.6% on the 3rd day, and the hematoma dissipation rate on the 7th day was 33.5%. The hematoma dissipation rate in the minimally invasive group was higher than that in the conservative treatment group on the 3rd and 7th day, and the difference was statistically significant (*P* < 0.05).  Figure 2 is comparison of hematoma clearance rate between the two groups on the 3rd and 7th day after operation.

### 3.5. Volume Comparison of Craniocerebral Hematoma between the Two Groups

The volume of craniocerebral hematoma was compared between the two groups at admission, the third day after operation, and the seventh day after operation. The results are shown in Figure 3. It was found that there was no significant difference in hematoma volume between minimally invasive group and conservative group at admission and on the 7th day after operation. On the 3rd day after operation, the hematoma volume of minimally invasive group was 16.5 ± 2.4 mL and that of conservative group was 27.4 ± 1.8 mL. There was significant difference between the two groups (*P* < 0.05). Moreover, through CT scanning, it was found that the hematoma volume of minimally invasive group and conservative group was significantly smaller than that of admission on the third day after operation, but the reduction degree of minimally invasive group was higher than that of conservative group, as shown in Figure 4.

### 3.6. Evaluation Indexes of Prognosis of Patients in the Two Groups

The prognosis of the two groups was evaluated by MRS score and ADL score. In this study, MRS score is ≤2, ADL score is grade I-II (70∼100), and the prognosis is good. The results are shown in Figure 5. There were 22 patients with good MRS prognosis in minimally invasive group, accounting for 73.3%, and 7 patients with good MRS prognosis in conservative group, accounting for 23.3%. There were 24 patients in the minimally invasive group with good ADL score prognosis, accounting for 80%, and 11 patients in the conservative group with good ADL score prognosis, accounting for 55%. It is found from the figure that the proportions of patients with MRS ≤2 and ADL grade I-II in the minimally invasive group are more than those in the conservative group. There was significant difference in the total scores of MRS and ADL between the two groups (*P* < 0.05).

## 4. Discussion

In China, cerebral hemorrhage patients account for about 48% of cardiovascular and cerebrovascular disease cases. Because of the rapid onset of cerebral hemorrhage and the critical condition at the time of onset, the annual mortality of cerebrovascular patients in China has reached 55% [13–15]. Epidemiological studies on cerebral hemorrhage in China show that the incidence rate of cerebral hemorrhage has exceeded 800 thousand. The age of onset is usually around 60 years, and the male patients aged 61∼70 are more than the female patients of the same age. The age group of the patients in this age group accounted for 31% of the total population [16–18].

At present, many researches apply intelligent algorithms to medical image processing. For example, Hu et al. [19] realized the processing of brain disease images by using fuzzy system. Li et al. [20] realized the research of medical image fusion based on deep learning algorithm. The classical unsupervised learning algorithm is clustering algorithm, and *K*-means clustering algorithm is commonly used in clustering algorithm. It is a clustering algorithm based on Euclidean distance. The basic principle is to use Euclidean distance to cluster the samples in the space as the cluster center and update the values of each center step by step through continuous iterative method, so as to output the best results. It has been found that the fuzzy *K*-means clustering algorithm can effectively divide the gray matter, cerebrospinal fluid, and white matter in the magnetic resonance brain image [21]. It is found that, compared with the two-dimensional maximum entropy algorithm, the *K*-means clustering algorithm has high quality and short average segmentation time for CT images of patients with cerebral hemorrhage.

The main pathogenesis of cerebral hemorrhage is the formation of hematoma in the brain. Hematoma will always exist in the brain. The sterile products of hematoma have toxic reactions to brain tissue. Toxic substances induce changes in the elasticity of cerebral vascular wall, resulting in cell edema and elevated intracranial pressure. The existence of hematoma bleeding points will destroy normal neural function. This study found that the hematoma volume of minimally invasive group was significantly smaller than that of conservative group on the third day after operation. Through CT examination, the hematoma volume of minimally invasive group and conservative group was significantly smaller than that of admission on the third day after operation, but the reduction degree of minimally invasive group was higher than that of conservative group. The hematoma dissipation rate of minimally invasive group on the third day after operation was 48.9%, and the hematoma clearance rate on the seventh day was 83.6%. Both results were higher than that of conservative treatment group at 16.6% on the third day and 33.5% on the seventh day.

For the treatment of cerebral hemorrhage, conservative drug treatment and minimally invasive hematoma debridement are often used in clinics. For elderly patients with cerebral hemorrhage, traditional craniotomy is not the best treatment. Compared with conservative drug treatment, minimally invasive puncture drainage has better therapeutic effect, is suitable for most patients, and has a better prognosis [22]. The study also found that the length of stay in the minimally invasive group was 10 ± 1.2 days and that in the conservative group was 18 ± 2.4 days. The length of stay in the minimally invasive group was significantly longer than that in the conservative group (*P* < 0.05). The total incidence rate of complications in the minimally invasive group was 10%, lower than that in the conservative group (25%) (*P* < 0.05). Based on this, it is suggested that minimally invasive puncture drainage can effectively and quickly remove craniocerebral hematoma, alleviate the increase of intracranial pressure caused by hematoma, and reduce the occurrence of complications [23].

This study found that the proportion of patients with good MRS score prognosis in the minimally invasive group was 3.15 times that in the conservative group. The ADL score of minimally invasive group was 1.6 times that of conservative group, and there was significant difference in the total score between the two groups (*P* < 0.05). It is proved that, compared with conservative treatment, minimally invasive surgery can significantly reduce the incidence rate of complications, shorten the length of stay, reduce the volume of hematoma, accelerate the evacuation of hematoma, improve the neurological function recovery and daily living ability of patients with cerebral hemorrhage, and greatly help the prognosis of patients with cerebral hemorrhage.

## 5. Conclusion

Minimally invasive puncture drainage is better than conservative treatment in the clearance of hematoma, which is conducive to the recovery of neurological function and daily life of patients with cerebral hemorrhage and is of great help to the prognosis of patients.

## Figures and Tables

**Figure 1:** Segmentation results of CT images by two algorithms: (a) the original CT images of patients with cerebral hemorrhage; (b) the lesion result segmented by two-dimensional maximum entropy algorithm; (c) the segmentation results of *K*-means clustering algorithm.

**Figure 2:** Comparison of hematoma clearance rate between the two groups on the 3rd and 7th day after operation: (a) the comparison result of hematoma clearance on the 3rd day; (b) the comparison result of hematoma clearance on the 7th day.

**Figure 3:** Comparison of hematoma volume between the two groups: (a) the hematoma volume of the two groups at admission; (b) the hematoma volume of the two groups on the 3rd day after operation; (c) the hematoma volume of the two groups on the 7th day after operation; there was significant difference between groups, ^*∗*^*p* < 0.05.

**Figure 4:** CT images of hematoma at admission and on the third day in the two groups: (a) the CT of hematoma at admission in the minimally invasive group; (b) hematoma CT on the 3rd day after operation in minimally invasive group; (c) the CT of hematoma at admission in the conservative group; (d) the CT of hematoma on the 3rd day after operation in the conservative group.

**Figure 5:** MRS score and ADL score results of the two groups: (a) the proportion of patients with MRS score ≤2 points in the two groups; (b) the proportion of patients with MRS score >3 in the two groups; (c) the proportion of patients with ADL score in stage I∼II; (d) the proportion of patients with stage III-IV in the two groups; (e) represents the MRS total score of the two groups; (f) the total ADL score of the two groups. The difference between groups was statistically significant, ^*∗*^*p* < 0.05.

**Table 1:** MRS and ADL scores.

Symptom	MRS	ADL
Completely healthy	0	I
Some mild to moderate symptoms	1	II
Having severe symptoms	2	III
Plant survival or death	3	IV

**Table 2:** Basic data of two groups of patients.

Project	Grade	Number of patients	
		Minimally invasive group	Conservative group
Age	<43	9	13
	≥43	11	17

Gender	Men	18	11
	Women	12	9

Level of consciousness	Completely clear	3	2
	Lethargy	11	5
	Coma	16	13

Onset time/h		8.2 ± 3.1	7.9 ± 2.5
History of hypertension/years		7.62 ± 4.24	7.03 ± 2.75
Bleeding volume/ml		27 ± 3.27	27 ± 2.26

**Table 3:** Comparison results of complications and length of stay between the two groups.

Grouping	Complication/*n*				Length of hospital stay/d
	Intracranial infection	Lung infection	Bleeding	Total incidence (%)	
Minimally invasive group	0	1	2	3 (10%)	10 ± 1.2
Conservative group	1	2	2	5 (25%)	18 ± 2.4
*P* value	0.187	0.095	0.621	0.027	0.003

## Data Availability

The simulation experiment data used to support the findings of this study are available from the corresponding author upon request.
